The article "A Search Method for Optimal Band Combination of Hyperspectral Imagery Based on Two Layers Selection Strategy" was published in 2021. Journal: Comput Intell Neurosci.

# A Search Method for Optimal Band Combination of Hyperspectral Imagery Based on Two Layers Selection Strategy

**DOI:** 10.1155/2021/5592323

**Published:** 2021-06-22

**Authors:** Nian Chen, Kezhong Lu, Hao Zhou

**Affiliations:** ^1^School of Big Data and Artificial Intelligence, Chizhou University, Chizhou 247000, China; ^2^College of Computer Science and Technology, Nanjing University of Aeronautics and Astronautics, Nanjing 211106, China; ^3^College of Computer and Information Science, Southwest University, Chongqing 400715, China

## Abstract

A band selection method based on two layers selection (TLS) strategy, which forms an optimal subset from all-bands set to reconstitute the original hyperspectral imagery (HSI) and aims to cost a fewer bands for better performances, is proposed in this paper. As its name implies, TLS picks out the bands with low correlation and a large amount of information into the target set to reach dimensionality reduction for HSI via two phases. Specifically, the fast density peaks clustering (FDPC) algorithm is used to select the most representative node in each cluster to build a candidate set at first. During the implementation, we normalize the local density and relative distance and utilize the dynamic cutoff distance to weaken the influence of density so that the selection is more likely to be carried out in scattered clusters than in high-density ones. After that, we conduct a further selection in the candidate set using mRMR strategy and comprehensive measurement of information (CMI), and the eventual winners will be selected into the target set. Compared with other six state-of-the-art unsupervised algorithms on three real-world HSI data sets, the results show that TLS can group the bands with lower correlation and richer information and has obvious advantages in indicators of overall accuracy (OA), average accuracy (AA), and Kappa coefficient.

## 1. Introduction

Hyperspectral imagery (HSI) is a combination of computer generated imagery (CGI) and spectral detection technology, and it can help us analyze the characteristics of objects without direct contact. Since each pixel in HSI has both plane coordinate and spectral information, we usually describe HSI as a three-dimensional cube; that is, on the spectral axis, each band corresponds to a 2D image. Due to the different degree of absorption and reflection of object surface against electromagnetic waves with various wavelengths, as well as the continuous accuracy improvement of spectral acquisition instruments, spectra are distributed on hundreds of narrow bands (generally bandwidth less than 10 nm) continuously. Up to now, HSIs obtained via remote sensing mapping are widely applied for data analyses in many application fields, such as mineral exploration [1], environmental and atmospheric monitoring [2, 3], and agricultural information services [4]. Compared with color image and multispectral image, more information can be recorded in HSI because of its high resolution, which is very useful for targets classification. However, it also brings some technological obstacles such as high dimensionality and information redundancy owing to similar or overlapped bands. Existing research studies have shown that high correlations frequently appear in some adjacent bands that probably cause the “Hughes phenomenon” [5]. Therefore, we always preprocess the spectrum before classification, including noise removed and redundancy reduction, which can effectively cut down the operation costs and improve the processing speed on the premise of maintaining accuracy of image recognition.

There are two approaches to achieve dimensionality reduction for HSI, i.e., band extraction and band selection (BS) [6, 7]. The former projects the all-bands into low dimensional subspace to form a simplified image; however, it may lead inherent feature of information to change. Some recent technologies include singular spectrum analysis [8], sparse representation [9], and stacked auto-encoders [10]. In essence, BS is a combined optimization problem; that is, we should find out a band combination with rich information, low correlation, and good discrimination via the evaluation criteria function. Whatever method is adopted, it is difficult to increase speed and accuracy simultaneously, so a common practice is that improve the efficiency of dimensionality reduction by optimizing some existent algorithms.

In this paper, our main contributions are summarized as follows. (1) Strategy of two layers selection is proposed for generating an optimal band combination. Specifically, we build a candidate set U using the bands selected by FDPC at first, and then spectral analyses are conducted to choose the high-quality elements from U, where we take not only information contained in a single band but also correlation of interband into consideration. (2) We put forward a new information evaluation method called comprehensive measurement of information (CMI), and by introducing the standard deviation and k-neighbors average similarity, both individual information and correlations among each other are considered synthetically. (3) Inspired by the idea of the greedy algorithm, we adopt the mRMR method to enrich the target set iteratively that can minimize redundancy and maximize representativeness.

The remaining sections are organized as follows. In Section 2, we will introduce some related research work about BS technologies in recent years. In the following section, principles of FDPC and information analysis as well as implementation flow of mRMR will be presented in detail. In Section 4, we state concretely how to build an optimal subset to replace the original spectrum via the TLS algorithm. A series of experiments and comparative analyses for results will be conducted to prove the efficiency of the proposed algorithm, and we arrange these in Section 5. In the last section, some conclusions will be given.

## 2. Related Work

As mentioned previously, it is an effective way to reduce the spectral dimensions of HSI via BS because this preprocessing can remove the redundant parts contained in the original spectrum, which is beneficial to decreasing the storage and computing consumption for subsequent image procession. If we have grasped the facts that various objects reflect against the electromagnetic waves, establishing an object-spectrum dictionary can guide us to select bands accurately; however, it is time-consuming, costly, and even impossible to get them in many cases. Unsupervised methods can well adapt to various application scenarios, which just make full use of the band distribution and interband relationship. At present, unsupervised BS is mainly categorized into ranking-based method, searching-based method, sparsity-based method, clustering-based method, and so on.

### 2.1. Unsupervised Band Selection Methods

For a long time, the research studies related to BS mainly focus on two themes. One is the selection algorithm that is commonly designed by using idea of supervised, semisupervised, or unsupervised method, and the other is the output evaluation criterion which is adopted to measure the performance of an algorithm. According to the needs of discussion, we briefly introduce some unsupervised methods, as well as corresponding algorithms used in Section 5.

The ranking-based method evaluates the importance of a band by using a criterion and employs top-ranked ones instead of all-bands to represent HSI. Clearly, this method can find out most discriminative bands, while the high correlation is inevitable owing to differences between each other neglected. Constrained band selection (CBS) [11] and maximum variance principal component analysis (MVPCA) [12] are both typical ranking-based algorithms. Compared with CBS, MVPCA is more sensitive to noise, so it should be used selectively according to the characteristics of data sets.

The searching-based method converts BS into an optimization problem of a given criterion and iteratively searches for the best bands to constitute a target set. For example, in [13], linear prediction (LP) is adopted to evaluate the similarity between a single band and other ones, and on this basis, the best band in current round is picked out. The sparsity-based method uses sparse representation or regression to reveal the information structure of a data set, and we select the representative bands by solving an optimization problem using sparsity constraints. The improved sparse subspace clustering (ISSC) algorithm [14] which will be employed for comparative analysis in Section 5is a sparse representation-based method.

Nodes belonged to the same cluster have similar features, so based on clustering, we select several exemplars to replace the entire cluster. Hierarchical-based clustering firstly initializes the whole set or a single node as a cluster and then groups the nodes by aggregation or splitting. Classical algorithms include WaLuDi [15], BIRCH [16], and CURE [17]. For the partition-based clustering algorithm, both number and centers of the clusters must be initialized in advance. We adjust the composition of each cluster by constantly updating the ownership of nodes until the stop condition is met. Some typical algorithms, such as *K*-means [18] and FCM [19], are widely applied in various classification applications. Observed from the perspective of geometric distribution, the high-density areas are separated by low-density ones, and each cluster is corresponding to a data subset with the maximum local density that can be connected. Therefore, the density-based algorithm can solve the classification problem for irregularly spatial distribution perfectly, and some algorithms, such as AP [20], DBSCAN [21], and FDPC [22], have shown good performances in nonspherical distribution clustering.

In the process of seeking a target set to reconstitute HSI, both initialization parameters and noise information impact greatly on the implementation effect. In many cases, the capability of an algorithm depends on initial parameters heavily, and the improper parameters may cause deviations between the clustering results and actual situations, even significant errors. Furthermore, during image acquisition, noises are generated inevitably owing to the environment or imaging equipment, which probably bring obstacles to subsequent processing. Usually, noise nodes are outliers with low density, so the density-based clustering algorithm has prominent advantage to noise recognition.

### 2.2. Fast Density Peaks Clustering

The FDPC algorithm was proposed by Rodriguez and Laio in 2014, which can obtain the globally optimal solution through a few parameters and simple process (no iteration required), and an obvious advantage compared with other clustering-based algorithms is that it can find arbitrary-shaped clusters, rather than just spherical regions. In the field of HSI processing, besides band selection [23], FDPC is also applied to superpixel segmentation [24]. Nevertheless, its performance still needs to be promoted, including computational complexity reduction, adaptive ability of parameters enhanced, and accuracy and robustness improved.

The time complexity of FDPC is O(n^2^) without considering dimensions, where *n* is the number of nodes. Accordingly, the algorithm is unsuitable for large-scale data clustering because of its high complexity. As improvements, researchers introduce parallel algorithms (e.g., EDDPC [25] and LSH-DDP [26]) or use grid treatment in advance (e.g., DGB [27], DPCG [28], and PDPC [29]) to accelerate it. For example, FastDPC-KNN [30] provides a solution, in which KNN is adopted to cooperate with FDPC, and the time complexity is reduced to O(n.log2^n^). It utilizes cover tree to speed up the calculation by distinguishing the type of peak density so as to avoid calculating the distance in the global range.

Parameter self-adaption (PS) is another important research issue for FDPC. Specifically, cutoff distance delimits the neighborhood size of each node that directly determines the statistical result of local density and also has a great influence on the composition of clusters. PS can cut down the probability of errors caused by experience setting, and it is more adaptable to various data scenarios. Researchers have employed some methods such as density estimation [31] and ADPC-KNN [32] to realize the PS.

## 3. Method and Strategy

### 3.1. FDPC for Candidate Set

FDPC is based on the following two assumptions. In each cluster, firstly, the density of a center is higher than that of the surrounding nodes, and secondly distance between the center and higher density node is relatively large. Moreover, there are two extremely important values in the algorithm, i.e., local density *ρ*and relative distance *δ*, and both of them depend on the similarity matrix *S*. A hyperspectral image *I* can be described in both spectral and geometric spaces, *I* = (*b*_1_, *b*_2_,…, *b*_*L*_) = (*x*_1_, *x*_2_,…, *x*_*N*_), where *L* and *N* are denoted as the number of bands and pixels, respectively. Thus, *b*_*l*_ = {*b*_*l*_^*i*^*|i* = 1,2,…, *N*} is the response of all pixels to *l*_th_ band, and *x*_*t*_ = {*x*_*t*_^*i*^*|i* = 1,2,…, *L*} is reflection of *t*_th_ pixel on different bands. Generally, we should build an initial similarity matrix *S* = *R*^*L*×*L*^ at first, and the similarity between b and *i* and *j* is expressed as the following equation:

(1) $$\begin{array}{c} S_{ij}={\left\|R_{i}-R_{j}\right\|}^{2}=\sum_{n=1}^{N}{\left(R_{ni}-R_{nj}\right)}^{2}. \end{array}$$

In practice, Gaussian kernel function *R*_*G*_(*x*, *y*) = exp(−‖*x* − *y*‖^2^/2*σ*^2^) is commonly applied to calculate Euclidian distance. In equation (2), *d*_*ij*_ is defined as the interband distance based on matrix*S*, and we obtain the correlation between the pairwise bands. Obviously, the closer two bands are, the higher redundancy is.

(2) $$\begin{array}{c} d_{ij}=\frac{\sqrt{S_{ij}}}{L}. \end{array}$$

Closely related to cutoff distance *d*_*c*_, the local density *ρ*_*i*_is defined as follows:

(3) $$\begin{array}{c} \rho_{i}=\sum_{j=1,j\neq i}^{L}\chi \left(d_{ij}-d_{c}\right),\\ \chi \left(x\right)=\left\{\begin{array}{c} 1,\;x\leq 0,\\ 0,\;x>0. \end{array}\right) \end{array}$$

A convenient and intuitive way to get *ρ*_*i*_ is that indicator function *χ* accumulates the nodes with Euclidean distances from *b*_*i*_ is less than *d*_*c*_. However, this approach does not distinguish the contribution of distance to density, and *ρ*_*i*_ increases by one as long as *d*_*ij*_ < *d*_*c*_. Hence, we also adopt Gaussian kernel function to overcome the limitation.

(4) $$\begin{array}{c} \rho_{i}=\sum_{j}\exp\left(-{\left(\frac{d_{ij}}{d_{c}}\right)}^{2}\right), \end{array}$$

*d*_*c*_ is the only parameter provided for human-machine interaction, and experience shows that the algorithm performs well when *d*_*c*_ is set to 1%-2% of all interband distances sorted in descending order. Inappropriate *d*_*c*_ may cause high overlap between clusters or produce a large number of meaningless clusters. Since FDPC is very sensitive to *d*_*c*_, we should set it precisely through some reasonable methods, e.g., PSO [33] and ADPclust [34], rather than relying on the empirical values. In Section 4.2, we determine *d*_*c*_ according to the number of required bands.

Next, we give the definition of *δ*_*i*_ as the following equation:

(5) $$\begin{array}{c} \delta_{i}=\left\{\begin{array}{cc} \underset{j:\rho_{i}<\rho_{j}}{\min}d_{ij}, & \exists j\text{ s}.\text{t}.\;\rho_{i}<\rho_{j}\\ \underset{j}{\max}d_{ij}, & \text{otherwise,} \end{array}\right) \end{array}$$

*δ*_*i*_ is the distance between *b*_*i*_ and the node farthest from it, only when *b*_*i*_ has the maximum local density. More generally, there are several nodes with higher density around *b*_*i*_; the distance between it and the nearest node is taken as *δ*_*i*_. After *ρ* and *δ* of all nodes are obtained, we establish the decision graph to describe them. In Figure 1(b), the nodes that can act as cluster centers are usual outliers; for example, node 1 has the largest projection values on two-dimensional axis, which means that it has both highest local density and sufficient intercluster spacing.

However, most of the remaining nodes are concentrated near the bottom of graph with small *δ* (region B), which indicates that they are grouped around the high-density nodes and have less power to be independent centers. In addition, FDPC has strong noise detection capability, and it can help us eliminate interference bands before BS. In Figure 1(b), the nodes near the vertical axis are probably labeled as noise ones, e.g., node 27 and 28.

For each *b*_*i*_, we utilize inner product *γ*_*i*_ = *ρ*_*i*_ × *δ*_*i*_ to integrate density and distance at first and sort *γ* in descending order for getting a priority sequence *γ*_1_ > *γ*_2_ > ⋯>*γ*_*m*_ > *γ*_*m*+1_ > ⋯>*γ*_*L*_. On this basis, we select *m* top-ranked bands, i.e., {*b*_spt(*γ*_1_)_, *b*_spt(*γ*_2_)_,…, *b*_spt(*γ*_*m*_)_} to form a candidate set U, where spt(*γ*_*i*_) is the subscript of band corresponding to *γ*_*i*_ and *m* is the number of required bands. The outputs of FDPC are all exemplars in each cluster, and the vital information is maintained accordingly. However, some bands that can provide more information for classifier are probably not picked out, such as boundary ones, because FDPC is more likely to select in high-density regions rather than low-density ones. Hence, based on the candidate set, we must conduct further analysis from the perspective of spectral information.

### 3.2. Layer 2 Selection for Target Set

In this paper, we analyze the amount of information (AoI) and band correlation as foundation and integrate them to evaluate information comprehensively. As stated in the last section, the bands selected by FDPC are already representative, whereas it is one-sided owing to just from the view of spatial position which implies that less, similar, or overlapped information may still exist in candidate set.

#### 3.2.1. Comprehensive Measurement of Information

Shannon entropy is a common index to measure event uncertainty, and researchers usually employ it to distinguish the AoI contained in a band. It is generally believed that an event with large entropy corresponds to strong uncertainty, which means that more information can be provided for judgement. Assuming that the band *b*_*i*_  gets different values with various probabilities, its Shannon entropy is defined as equation (6), where *b*_*ik*_ is the *k*_*th*_ possible value of *b*_*i*_.

(6) $$\begin{array}{c} H\left(b_{i}\right)=-\sum_{k}p\left(b_{ik}\right)lb\left(p\left(b_{ik}\right)\right). \end{array}$$

The standard deviation is another way to measure AoI, and it reflects the uncertainty through the difference between a set of data and its mean value, as defined in the following equation:

(7) $$\begin{array}{c} \mu_{i}=\sqrt{\frac{\sum_{k=1}^{N}{\left(b_{ik}-{\bar{b}}_{i}\right)}^{2}}{N}}, \end{array}$$

where $\bar{b_{i}}$is the mean value of *b*_*ik*_. Apparently, greater *μ*_*i*_ corresponds to large AoI.

It is improper to consider AoI in a single band alone, but ignore the relationships among them because high information correlation between adjacent bands is also very common, just like spatial redundancy.

Hence, we put forward CMI to reevaluate information situation for a band by taking both AoI and information redundancy into account comprehensively.

(8) $$\begin{array}{c} \text{CMI}\left(b_{i}\right)=\frac{\mu_{i}}{\bar{\varphi_{i}}}=\frac{\mu_{i}}{\left(\sum_{j=i-\left(h/2\right)}^{i+\left(h/2\right)}\varphi_{i,j}\right)/h}. \end{array}$$

The correlation between *b*_*i*_ and its *h*-neighbors is measured by average similarity $\bar{\varphi_{i}}$, where *φ*_*i*,*j*_ ∈ (0,1) is correlation coefficient between adjacent bands and *h* is an even number. For example, when *h* = 2, we judge the information independence of *b*_*i*_ via average similarity on pairs of (*b*_*i*−1_, *b*_*i*_ , *b*_*i*+1_), which is called the nearest neighbor metric. In general, we get $\bar{\varphi_{i}}$ in a wider neighborhood by appropriately increasing *h* because we cannot guarantee that *φ*_*i*,*i*+1_ is always greater than *φ*_*i*,*i*+2_. However, the probability of information redundancy between bands with large label difference is very small, so excessive *h* may cause meaningless computation.

According to equation (8), if *b*_*i*_ is what we are looking for, it should have either a large *μ*_*i*_ or a small $\bar{\varphi_{i}}$ or both. Hence, it can prevent bands with high information redundancy from being selected via CMI.

#### 3.2.2. Further Selection Employed mRMR

The abbreviation mRMR denotes maximum representativeness and minimum redundancy.*ρ*has a larger weight because of measurement scale during the implementation of FDPC, so the targets are most probably generated in the high-density regions. In Figure 1(b), if we want to select more from region B, the results must be the neighbors of node 1 instead of any node else. Clearly, FDPC guarantees the representativeness of candidate set but inclines to cause redundancy, so based on its outputs, we employ mRMR strategy to conduct a further filter.

Let *U* = {*b*_1_, *b*_2_,…, *b*_*m*_} be the candidate set, and target set and residual set are denoted as *U*_*t*_ and *U*_*r*_, respectively; *U* = *U*_*t*_ ∪  *U*_*r*_. Supposing that *k* (*k* ≥ 1) bands have already existed in *U*_*t*_, if the (*k* + 1) th band is required from *U*_*r*_to enrich *U*_*t*_, the best one should satisfy the following conditions. (1) Lowest correlation within *U*_*t*_, that is, the average distance from it to every element in *U*_*t*_ is farthest; (2) Highest similarity with *U*_*r*_, which indicates that it has the most power to represent other bands in *U*_*r*_. According to formula (9), we select the most appropriate *b*_*i*_ ∈ *U*_*r*_.

(9) $$\begin{array}{c} \underset{b_{i}\in U_{r}}{\arg\max}\left(\frac{1}{k}\underset{b_{j}\in U_{t}}{\sum }d_{i,j}-\frac{1}{m-k}\underset{b_{j}\in U_{r}}{\sum }d_{i,j}\right). \end{array}$$

Motivated by above descriptions, taking AoI and information correlation into account simultaneously as formula (10), we get the target set with strong representativeness, good discrimination, and low redundancy to reach dimensionality reduction for HSI.

(10) $$\begin{array}{c} \underset{b_{i}\in U_{r}}{\arg\max}\left[\left(\frac{1}{k}\underset{b_{j}\in U_{t}}{\sum }d_{i,j}-\frac{1}{m-k}\underset{b_{j}\in U_{r}}{\sum }d_{i,j}\right)\times \text{CMI}\left(b_{i}\right)\right]. \end{array}$$

## 4. TLS Algorithm

### 4.1. Implementation Flow

TLS integrates spatial position, information contained in a single band, and correlation between each other to evaluate the importance of a band, so it is suitable for spectral dimensionality reduction because of the comprehensiveness of its outputs.

In this section, we explain how TLS works. As the preliminary BS (layer 1 selection), FDPC prioritizes the bands firstly and selects the top-ranked ones to establish *U*. In layer 2, we make some relevant initialization for preparation, *U*_*t*_ = {*b*_spt(*γ*_1_)_}, *U*_*r*_ = {*b*_*j*_*|j* = spt(*γ*_2_), spt(*γ*_3_),…, spt(*γ*_*m*_)}, and score for each band in *U* by using CMI index. In current round, the most valuable band *b*_*p*_ satisfied formula (10) is picked out to join *U*_*t*_, and those ones that have approximate information to *b*_*p*_ will be removed from *U*_*r*_. Iterate until *U*_*r*_ = ∅, and the informative and low information-redundancy band combination is built.

We give the technology roadmap of TLS as Figure 2.

TLS filters the redundant information bands via threshold *λ*. According to equation (8), *b*_*p*_ becomes the winner in a certain selection round only when it has both rich AoI and strong information independence. For each *b*_*q*_ ∈ *U*_*r*_, *p* ≠ *q*, if *φ*_*p*,*q*_ > *λ*, we take *b*_*q*_out of *U*_*r*_owing to its high correlation. We state the implementation flow of TLS in Algorithm 1and put some related explanations and analyses in Section 4.2and 4.3.

### 4.2. Normalization and Parameter Initialization

As mentioned previously, different metrics cause that *ρ*has a heavy impact on prioritization, and bands with high-densities are more attractive to FDPC. As a direct improvement, both *ρ*and *δ*are normalized to interval (0, 1).

(11) $$\begin{array}{c} {\tilde{\rho }}_{i}=\frac{\left(\rho_{i}-\rho_{\min}\right)}{\left(\rho_{\max}-\rho_{\min}\right)},\\ {\tilde{\delta }}_{i}=\frac{\left(\delta_{i}-\delta_{\min}\right)}{\left(\delta_{\max}-\delta_{\min}\right)}. \end{array}$$

In addition, we also reduce the influence of *ρ*by adjusting *d*_*c*_dynamically so that the probability of selecting in the low-density regions increases gradually. Improper *d*_*c*_ may lead to algorithm failure, even domino effect happened and cannot be corrected by itself. For the sake of simplicity, the empirical method sets *d*_*c*_with fixed size; however, it is inefficient when dealing with high-dimensional data or fake peaks.

In order to make the density value relatively accurate, it ought to be avoided as much as possible that a band appears in different neighborhood repeatedly. Hence, we deem that *d*_*c*_ should not be fixed but change dynamically corresponding to *m*, shown as the following equation:

(12) $$\begin{array}{c} d_{c}=\alpha \times d_{c-0}\\ =\log_{2}\frac{L}{m}\times d_{c-0}, \end{array}$$

where *d*_*c*−0_ is the initial value of cutoff distance. With the increase in *m*, *d*_*c*_ keeps getting smaller, and the situation that a band belongs to different density neighborhood will gradually disappear. Usually, *m* < (*L*/2), and *d*_*c*−0_ is multiplied by a coefficient *α*to determine *d*_*c*_. In extreme case, if each node corresponds to a cluster, i.e., *m* = *L*, we get *d*_*c*_ = 0.

### 4.3. Performance Analysis to TLS

The time complexity of FDPC is *O*(*N* × *L*^2^), which is mainly the time consumption of building similarity matrix. On this basis, TLS increases the cost of acquiring CMI of each band (linear complexity *O*(*m* × *N*) and iteratively generating the target set *O*(*m* × *N*). Therefore, in the field of dimensionality reduction to HSI, the time complexity of TLS is *O*(*N* × (*L*^2^ + *m*)) which affects the real-time performance when dealing with high-resolution images.

Besides high time complexity, TLS also needs to initialize *m* in advance because it has no ability to automatically configure the number of clusters according to the data distribution. In layer 1, no peak or fake peak will cause the proposed algorithm invalid, for the hypothesis that makes FDPC work does not hold. In addition, the outputs of mRMR are not back-traceable, which implies that it cannot be deleted if a band has been selected into the target set.

In conclusion, the distinct advantage is that TLS can find out a more effective band combination in the condition of using the same *m* with others. Clearly, TLS not only inherits the characteristics of FDPC, such as good at exemplar selection, noise insensitivity, and no initialization to cluster center, but also makes information to be an important reference by using CMI.

## 5. Experiment and Discussion

In this section, a series of comparative experiments have been designed and implemented on three HSI data sets, and the capability comparisons of TLS and other state-of-the-art algorithms using OA, AA, and Kappa coefficient are followed. Analyses and discussions are carried out in three aspects: (1) the difference of band distribution formed by various algorithms; (2) influence of number of the selected bands on HSI performance; and (3) influence of other factors, such as classification model and data set, on the performance of the algorithms. Before the experiments, the relevant contents should be introduced firstly, including data sets, algorithm competitors, classifiers for validation, and indicators for capability comparison.

### 5.1. Preparation for Experiments

#### 5.1.1. Data Sets

Three real-world HSI data sets which are derived from remote sensing images, i.e., Indian Pines, Pavia University (PaviaU), and Salinas are used for experiments. The essential information about them is briefly described in Table 1.

As universal data sets, there are some common characteristics with them. First of all, pixels of land cover that belong to the same class have the similar features, whereas the spectra corresponding to distinct classes are obviously different, which is very suitable for BS by clustering methods. Secondly, the distribution of pixels among classes is inhomogeneous and even most pixels of HSI are concentrated in a few bands, as shown in Figure 3. Finally, some contaminated bands have been removed to ensure the validity of the data; for example, 16 bands disturbed by external circumstances in Indian Pines, which are numbered 104–108, 150–163 and 220, are cleared beforehand.

#### 5.1.2. Basic Setup for Experiment

In order to verify the effectiveness of TLS, in this paper, MVPCA [12], WaLuDi [15], DBSCAN [21], FDPC [22], LP [13], and ISSC [14] algorithms are applied to reconstitute HSIs as competitors, respectively.

We train KNN (*K* = 5) and SVM (RBF kernel function) models with labeled samples in advance, and the classifiers have stronger generalization ability after sufficient experiences mastered. Due to the uncertainty of individual result, we take the average of 10 rounds as finals using cross-validation so as to make the outputs of algorithms more referable and convincing. In Indian Pines/PaviaU/Salinas, 30%/10%/10% pixels in every class are for classifiers learning and 10%/5%/5% ones are for tests during each round.

For a specific data set, we set the ranges of parameters and thresholds for testing, and the values corresponding to the best results are adopted. The detailed settings are as follows: *d*_*c*−0_ = min*d*_*ij*_, *m* < (*L*/2), *h* ∈ [2,8], *λ* = *c* × max*φ*_*i*,*j*_, and *c* ∈ [0.8, 0.95].

#### 5.1.3. Performance Indicators

OA, AA, and Kappa coefficient are commonly used as indicators to evaluate classification effect based on confusion matrix. OA represents the ratio of number of correctly classified pixels to the total; however, it cannot show the real situation when the class-scale difference is relatively large. As a more reasonable metric, AA reflects the recognition accuracy on a single class. Kappa coefficient is usually employed for consistency check, and in general, a larger Kappa coefficient means that the prediction results are more consistent with the ground truths. Specifically, conclusion is substantial when 0.8 > Kappa > 0.6, while Kappa ≥ 0.8 corresponds to perfect matching.

### 5.2. Results Analysis and Discussion

#### 5.2.1. Distribution of Algorithm Outputs

As mentioned in Section 5.1.2, seven algorithms are adopted to select bands, representing the original image with reduced spectral dimensions. For example, the results of 10 bands selected in Indian Pines are shown in Figure 4, from which we can observe the band distribution and redundancy intuitively.

Obviously, the redundancy produced by MVPCA is highest among all the employed algorithms, and most of selected bands are concentrated in the interval [120, 140]. As stated in Section 2, the ranking-based algorithm can find out critical bands efficiently by prioritizing, while it probably results in high redundancy and low discrimination because of correlation between the bands neglected. There are no significant differences in the performance of remaining algorithms although ideas they adopted are not exactly the same. The selection results are not uniformly distributed in entire band interval, and concentration may appear in some local intervals. In Figure 4, different algorithms will conduct selections in the same interval, which means that the attractiveness of interval with remarkable characteristics to various algorithms is similar, but the specific output within an interval may be different. Nevertheless, the dispersion of bands selected by TLS in global range is still better than that of some competitors because layer 2 plays an effective role. From the illustration, the concentrated bands appear in four/three intervals intuitively when we employ FDPC/DBSCAN, whereas they appear in just two if WaLuDi/LP/ISSC/TLS is used.

#### 5.2.2. Accuracy and Consistency Check

*Comparison of Accuracy Index*. As illustrated in Figures 5–7, we conclude common characteristics at first. No matter what algorithm or data set is employed, the improvement of OA is always synchronized with the increase in *m*. Nevertheless, the band contributions to classifier decrease gradually, which implies that excessive selections have no great significance for the evolution of classifier parameter. As Figure 5(b), OA of each algorithm except MVPCA has been improved by about 20% which is brought by the increase in *m* from 6 to 30; however, if we raise the number to 36 or 42, OAs are maintained at the current level and the classification capability has not gone better obviously.

Moreover, the effects of the reduced sets formed by different algorithms to image recognition are unstable, which depends on both the classifier model and data set. Intuitively, OA of the SVM model is higher than that of KNN in Indian Pines significantly, while the performances of two classifiers are not widely different in PaviaU and Salinas. From the view of the model, SVM seeks a hyperplane to maximize the margin between two classes by learning the experiences provided by support vectors, and it has good generalization power, as well as strong ability of noise resistance. Differently, KNN uses the nearest neighbors voting method to determine the class attribution of a sample, and its accuracy is slightly lower than SVM. On the other hand, the capability of the same algorithm may be diverse when dealing with different data set, and for each algorithm, OAs in PaviaU and Salinas are superior to those in Indian pines. Evidently, there are several small-scale classes in Indian Pines, even three ones with less than 50 samples (Figure 3(a)), and samples contained in these classes have high probabilities of misclassification that make OA declining.

According to the number of available bands *L*, we take *m* = (1/5)*L*as required number (40 bands from Indian Pines and Salinas and 20 bands from PaviaU), and the accuracy of individual class, AA, and OA of algorithm is shown in Tables 2–4. In each table, we notice the following facts. Firstly, whatever algorithm is employed, the recognition accuracies on most small-scale classes are relatively lower (such as grass-pasture-mowed, oats, buildings-grass-trees-drives in Table 2, gravel in Table 3, and lettuce-romaine-6wk in Table 4), but there are exceptions (such as wheat in Table 2and shadows in Table 3). This may be caused by over-fit that classifier takes OA as the criterion to fit the samples on training set as much as possible. It will generate some false negative samples on the small-scale class during model training; in other words, some samples that originally belong to small-scale class are wrongly classified to large-scale one. Therefore, when the classification model is applied to test set, its generalization ability will decrease. Although AA can make up for this defect, the main way is to reserve an appropriate number of bands with high quality to promote the discrimination ability of classifier. Secondly, OA is larger than AA and the difference reflected in Indian Pines is more prominent. Compared with averaging accuracies of all classes, it can make smaller impact to accuracy if we use proportion of quantity. Finally, some algorithms perform well just on the specific classes (such as MVPCA on Alfalfa in Table 2and DBSCAN on self-blocking bricks in Table 3), which means that the effect of the algorithm relates not only to class scale but also to match degree to data distribution. Similarly, TLS is not superior to its competitors on some classes, such as Alfalfa and meadows, although it is the best on entire data set.

By comparing AA and OA, TLS has shown its superiority, and the performance of ISSC is closest to it. WaLuDi, DBSCAN, and FDPC have similar capabilities in the aspect of BS, whereas MVPCA and LP are relatively poor. The stability of an algorithm can be shown via variance, and a small variance corresponds to low volatility. In Tables 3and 4, the recognition accuracy of TLS on each class has the smallest change relative to the mean value, whereas its stability is second only to ISSC in Table 2.

In particular, if we want a rough recognition for HSI quickly, TLS can pick out a few high-quality bands to accelerate the training process of classifier. For example, in Figure 6(a), the accuracy of TLS exceeds 70% by training the SVM model with only 6 bands, which is about 5% higher than that of WaLuDi, LP, and FDPC. However, the advantage of TLS is gradually weakened along with more bands appended, and OA of various algorithms is quite close when *m* reaches a certain value.

*Comparison of Consistency Index*. In Table 5, Kappa coefficients of various algorithms with different *m* are all within the interval (0.7, 0.95), indicating that the classification results are highly consistent with the actual values in spite of only a part of ones utilized to represent the entire set. Similarly, Kappa curve is also proportional to the number of selected bands, while the rising speed slows down step by step. Moreover, observed from the classification model and data set, it is confirmed that SVM is more suitable for working on these data sets, and we can obtain higher Kappa coefficients when conducting experiments on PaviaU and Salinas owing to its relatively balanced pixel distribution compared with Indian Pines. From the aspect of the algorithm, TLS has stronger discrimination and can help the classifier to make more accurate judgement.

#### 5.2.3. Execution Time

In Section 4.3, we have analyzed the time complexity of TLS and pointed out that the algorithm has no advantage in execution speed. The running time of the algorithm is mainly dependent on the hardware configuration; however, data set and the number of selected bands will also affect it. In this paper, the experiments run on a Windows 10 computer with an Intel i5 Quad Core processor and 8 GB of random-access memory. The corresponding execution time of seven algorithms under different conditions is shown in Table 6.

According to the setting in Section 5.1.2, the number of samples used for experiments varies on different data sets, which is clearly reflected by the time consumed, so the execution time of all algorithms is longest in PaviaU accordingly. Besides that the speed of an algorithm is greatly impacted by its execution mode, and there is no doubt that sort/noniteration may cost less time than iteration. Hence, MVPCA takes the least amount of time followed by ISSC, FDPC, and DBSCAN in order. TLS is faster than LP, and the time consumed by the WaluDi is the longest.

## 6. Conclusion

In this paper, we propose a two layers selection (TLS) algorithm to establish a dimensionality-reduced band set for HSI. On the premise of keeping the basic features of the spectrum, the bands with strong discrimination, low redundancy, and high information are picked out to complete the image reconstitution, and TLS achieves this goal through two phases. First, we employ the FDPC algorithm to sort the inner products of the local density and relative distance of all nodes in the all-bands set aiming at building a priority sequence, and the bands corresponding to top-ranks are collected into the candidate set. Owing to great influence of local density on FDPC outputs, we utilize methods of normalization and dynamic cutoff distance to realize the cherry-pick in scattered low-density regions as much as possible. After getting CMI, mRMR is adopted to group the bands that meet the given requirements in candidate set into the target set iteratively. In order to verify the effectiveness of TLS, six state-of-the-art algorithms are used as competitors to carry out experiments on three remote sensing image data sets. The comparative results that use indicators of OA, AA, and Kappa coefficient show that the band combination created by TLS is optimal. Especially, if we want a classification model to achieve higher accuracy with less training cost, TLS provides an effective way to cut down the dimensions of samples. Besides HSI processing, it also fits some applications where the sample has two or more types of features so that the hierarchical selection can be implemented.

Although lots of work has been done to improve the capability of the BS method, there are still many technical obstacles that need to be overcome in the future. Henceforth, the theory research studies will mainly focus on how to cut down the complexity of algorithms and improve their accuracy and robustness. Meanwhile, enhancing the adaptability to large-scale and high-dimensional data environment is also the direction of our innovation.

## Figures and Tables

**Figure 1:** Nodes distribution and decision graph: (a) the spatial distribution of nodes and (b) the decision graph corresponding to (a).

**Figure 2:** Technology roadmap of TLS. In layer 1, FDPC is employed to carry out preliminary selection from all-bands set to build a candidate set. In layer 2, AoI and correlation analyses are used to form optimal band combination.

**Figure 3:** Pixel distribution on different classes of three data sets. The subfigures are explained with the format of data set name, number of classes, and maximum difference ratio of interclass. (a) Indian Pines, 16, and 122.75 : 1; (b) PaviaU, 9, and 19.7 : 1; (c) Salinas, 16, and 12.3 : 1.

**Figure 4:** Comparison of band selection results with seven algorithms in Indian Pines.

**Figure 5:** In Indian Pines, OA curves correspond to different BS algorithms using (a) the SVM model and (b) the KNN model.

**Figure 6:** In PaviaU, OA curves correspond to different BS algorithms using (a) the SVM model and (b) the KNN model.

**Figure 7:** In Salinas, OA curves correspond to different BS algorithms using (a) the SVM model and (b) the KNN model.

**Algorithm 1:** Implementation flow of the TLS algorithm.

**Table 1:** Essential information of experimental data set.

Data set	Resolution	Pixels (background + object)	Bands	Available bands	Class
Indian Pines	145 × 145	21025 (10776 + 10249)	220	200	16
PaviaU	610 × 340	2207400 (2164624 + 42776)	115	103	9
Salinas	512 × 217	111104 (56975 + 54129)	224	204	16

**Table 2:** Classification accuracies (%) achieved using 40 selected bands in Indian Pines with KNN classifier.

Class	Algorithm						
	Accuracy (%)						
	MVPCA	WaLuDi	DBSCAN	FDPC	LP	ISSC	TLS
Alfalfa	66.8	54.6	50.5	39.2	33.7	34.2	45.4
Corn-notill	60.5	71.3	69.6	71	64.3	75.8	73.7
Corn-mintill	41.5	57.4	60	66.8	48.7	65.2	66.8
Corn	48.4	57.4	57.7	58.3	53.8	53.1	60.1
Grass-pasture	82.6	88.7	86.2	85	88.4	82.1	84.4
Grass-trees	93.1	94.5	95	94.3	93.3	96.7	96
Grass-pasture-mowed	45.2	44.8	42.1	37.3	71.7	92	45.2
Hay-windrowed	97.6	96.3	96.6	95.8	98.1	96.7	96.6
Oats	29.8	24.2	27	24.4	38.3	61.2	29.7
Soybean-notill	59.5	76.2	73.7	68.3	67.2	79.4	75.7
Soybean-mintill	77.4	79.3	81.5	82.6	82.9	82.5	84.2
Soybean-clean	43.1	69.6	71	72.2	58.9	83.3	72
Wheat	93	97.7	98.4	98.1	96.2	96.2	95.4
Woods	93.6	94.4	93.3	93.5	94.6	96.8	95.8
Buildings-grass-trees-drives	42.7	52.7	51.9	50.4	54.9	53.6	55.1
Stone-steel-towers	94.9	76.3	78.4	83.6	69.7	80.9	82.4

AA	66.8	70.9	70.6	70	69.7	76.9	72.4
OA	74	77.8	76.2	77.1	75.3	79.7	80.8
Variance	515.4	421.4	421.1	487.7	410.0	326.2	399.3

**Table 3:** Classification accuracies (%) achieved using 20 selected bands in PaviaU with SVM classifier.

Class	Algorithm						
	Accuracy (%)						
	MVPCA	WaLuDi	DBSCAN	FDPC	LP	ISSC	TLS
Asphalt	86.5	87.6	87.7	89.8	88.6	89.7	91.4
Meadows	96.4	96.8	96.2	94.8	94.7	98.1	96.6
Gravel	72.7	71.3	75.8	74.2	73.7	74.6	76.2
Trees	84.2	91.3	91	92.1	90.3	92.2	93.3
Painted metal sheets	99.1	99.4	99.4	97.8	97.3	98.2	99.1
Bare soil	53.2	82.5	81.5	82.4	80.4	82.8	83.5
Bitumen	79.8	83.8	81.7	76.6	80.1	82.7	83.3
Self-blocking bricks	83.4	85.2	86.3	83.8	82.4	83.6	84.9
Shadows	97.2	98.5	98.5	98	97.8	98.3	98.7

AA	83.6	88.4	88.6	87.7	87.3	88.9	89.6
OA	85.4	89.3	89.1	89.3	87.6	89.7	91.5
Variance	183.9	73.5	60.7	70.1	64.9	64.4	57.5

**Table 4:** Classification accuracies (%) achieved using 40 selected bands in Salinas with KNN classifier.

Class	Algorithm						
	Accuracy (%)						
	MVPCA	WaLuDi	DBSCAN	FDPC	LP	ISSC	TLS
Brocoli-green-weeds-1	83.4	84.5	83.2	82.7	82	84.4	84.7
Brocoli-green-weeds-2	88.8	92.3	90.2	94.2	89	91.7	91.4
Fallow	80.5	81.4	83.3	83.6	81.4	84.2	84.8
Fallow-rough-plow	76.4	80.5	79.2	77.8	79.6	80.4	81.1
Fallow-smooth	86.7	86.2	91.6	85	87.3	86.8	86.4
Stubble	92.8	93.1	89.6	91.6	89.2	90.4	88.7
Celery	87.7	89.1	92.4	92.8	90.3	92.2	87.4
Grapes-untrained	95.4	96.1	97.3	97	95.7	95.4	96.5
Soil-vinyard-develop	92.6	93.5	92.2	81.8	86.2	93.4	91.7
Corn-seneseed-green-weeds	86.9	89.5	86.2	90.3	84.2	86.3	87.7
Lettuce-romaine-4wk	75.4	79.2	78.5	80.4	75	79.3	79.7
Lettuce-romaine-5wk	81.6	83.2	83	84.4	81.2	81.6	84.8
Lettuce-romaine-6wk	74	72.6	72.3	76.2	73.6	75.3	75.5
Lettuce-romaine-7wk	73.2	76.3	74.8	75.5	74.6	75	77.4
Vinyard-untrained	95	95.3	94.7	95.2	91.2	95.6	96.2
Vinyard-vertical-trellis	80.4	80.7	81.7	81.6	76.7	81.5	82.3

AA	84.4	85.8	85.6	85.6	83.6	85.8	86.0
OA	87.5	89.2	89.1	89.8	88	89.2	90.8
Variance	52.0	47.9	50.1	45.6	41.4	42.7	34.7

**Table 5:** Kappa coefficients of algorithms under different conditions.

Algorithm		Data set					
		Kappa coefficient					
		Indian pines		PaviaU		Salinas	
		SVM	KNN	SVM	KNN	SVM	KNN
MVPCA	*m* = 12	0.723	0.708	0.782	0.796	0.77	0.762
	*m* = 18	0.771	0.756	0.846	0.853	0.853	0.867
	*m* = 24	0.806	0.782	0.873	0.872	0.893	0.901

WaLuDi	*m* = 12	0.714	0.702	0.824	0.829	0.816	0.814
	*m* = 18	0.787	0.771	0.881	0.867	0.875	0.86
	*m* = 24	0.821	0.804	0.918	0.89	0.91	0.893

DBSCAN	*m* = 12	0.726	0.71	0.797	0.784	0.813	0.806
	*m* = 18	0.783	0.773	0.872	0.861	0.878	0.88
	*m* = 24	0.822	0.818	0.905	0.903	0.911	0.917

FDPC	*m* = 12	0.72	0.732	0.804	0.796	0.822	0.808
	*m* = 18	0.782	0.797	0.852	0.865	0.885	0.86
	*m* = 24	0.817	0.83	0.897	0.902	0.907	0.902

LP	*m* = 12	0.716	0.704	0.803	0.78	0.797	0.804
	*m* = 18	0.768	0.76	0.854	0.841	0.853	0.86
	*m* = 24	0.811	0.797	0.87	0.882	0.88	0.894

ISSC	*m* = 12	0.736	0.715	0.845	0.84	0.833	0.838
	*m* = 18	0.792	0.773	0.893	0.903	0.887	0.891
	*m* = 24	0.83	0.81	0.921	0.926	0.92	0.923

TLS	*m* = 12	0.738	0.751	0.853	0.834	0.846	0.848
	*m* = 18	0.803	0.822	0.905	0.897	0.89	0.904
	*m* = 24	0.842	0.853	0.927	0.924	0.918	0.93

**Table 6:** The execution time of algorithms under different conditions.

Data set		Algorithm						
		Time (s)						
		MVPCA	WaLuDi	DBSCAN	FDPC	LP	ISSC	TLS
Indian Pines	*m* = 10	1.87	47.55	7.51	6.86	22.66	4.37	10.01
	*m* = 30	1.94	49.37	8.82	7.46	24.3	5.29	11.7
	*m* = 50	2.05	50.87	10.16	7.91	26.84	5.76	12.24

PaviaU	*m* = 10	5.76	93.22	13.46	13.7	42.26	10.44	17.66
	*m* = 30	5.93	95.63	15.28	15.26	44.63	12.26	19.44
	*m* = 50	6.14	96.87	16.9	15.53	45.58	12.81	20.63

Salinas	*m* = 10	3.61	71.46	10.33	9.74	29.84	8.86	13.3
	*m* = 30	3.83	72.73	11.97	10.67	31.4	10.42	15.54
	*m* = 50	4.04	74.3	13.42	10.93	32.66	11.34	16.62

## Data Availability

The data used to support the findings of this study are included within the paper.

## References

[1] Zadeh M. H., Tangestani M. H., Roldan F. V., Yusta I. (2014). Mineral exploration and alteration zone mapping using mixture tuned matched filtering approach on ASTER data at the central part of Dehaj-Sarduiyeh copper belt, SE Iran. *IEEE Journal of Selected Topics in Applied Earth Observations and Remote Sensing*.

[2] Gao B., Lu A., Pan Y. (2017). Additional sampling layout optimization method for environmental quality grade classifications of farmland soil. *IEEE Journal of Selected Topics in Applied Earth Observations and Remote Sensing*.

[3] Giardino C., Bresciani M., Valentini E. (2015). Airborne hyperspectral data to assess suspended particulate matter and aquatic vegetation in a shallow and turbid lake. *Remote Sensing of Environment*.

[4] Haboudane D., Miller J. R., Pattey E., Zarco-Tejada P. J., Strachan I. B. (2004). Hyperspectral vegetation indices and novel algorithms for predicting green LAI of crop canopies: modeling and validation in the context of precision agriculture. *Remote Sensing of Environment*.

[5] Hughes G. F. (1968). On the mean accuracy of statistical pattern recognizers. *IEEE Transaction on Information Theory*.

[6] Zhang W., Li X., Dou Y., Zhao L. (2018). A geometry-based band selection approach for hyperspectral image analysis. *IEEE Transaction on Geoscience and Remote Sensing*.

[7] Yuan Y., Lin J., Wang Q. (2016). Dual-clustering-based hyperspectral band selection by contextual analysis. *IEEE Transaction on Geoscience and Remote Sensing*.

[8] Zabalza J., Ren J., Zheng J. (2015). Novel two-dimensional singular spectrum analysis for effective feature extraction and data classification in hyperspectral imaging. *IEEE Transaction on Geoscience and Remote Sensing*.

[9] Qiao T., Yang Z., Ren J. (2018). Joint bilateral filtering and spectral similarity-based sparse representation: a generic framework for effective feature extraction and data classification in hyperspectral imaging. *Pattern Recognition*.

[10] Zabalza J., Ren J., Zheng J. (2016). Novel segmented stacked auto-encoder for effective dimensionality reduction and feature extraction in hyperspectral imaging. *Neurocomputing*.

[11] Chang C.-I., Wang S. (2006). Constrained band selection for hyperspectral imagery. *IEEE Transaction on Geoscience and Remote Sensing*.

[12] Chang C., Du Q., Sun T., Althouse M. L. G. (1999). A joint band prioritization and band-decorrelation approach to band selection for hyperspectral image classification. *IEEE Transaction on Geoscience and Remote Sensing*.

[13] Du Q., Yang H. (2008). Similarity-based unsupervised band selection for hyperspectral image analysis,. *IEEE Geoscience and Remote Sensing Letters*.

[14] Sun W., Zhang L., Du B., Li W., Lai Y. M. (2015). Band selection using improved sparse subspace clustering for hyperspectral imagery classification. *IEEE Journal of Selected Topics in Applied Earth Observations and Remote Sensing*.

[15] Us´o A. M., Pla F., Sotoca J. M., Garc´ıa-Sevilla P. (2007). Clustering-based hyperspectral band selection using information measures. *IEEE Transaction on Geoscience and Remote Sensing*.

[16] Zhang T., Ramkrishnan R., Livny M. (1996). Birch: An Efficient Data Clustering Method for Very Large Databases. *ACM Sigmod*.

[17] Guha S., Rastogi R., Kyuseok S. (2001). Cure: an efficient clustering algorithm for large databases. *Information Systems*.

[18] Jain A. K. (2010). Data clustering: 50 years beyond *K*-means. *Pattern Recognition Letters*.

[19] Xu R., Wunsch D. (2005). Survey of clustering algorithms. *IEEE Transaction on Neural Networks*.

[20] Freyb J., Dueck D. (2007). Clustering by passing messages between data points. *Science*.

[21] Ester M., Kriegel H., Sander J. A density-based algorithm for discovering clusters in large spatial databases with noise.

[22] Rodriguez A., Laio A. (2014). Clustering by fast search and find of density peaks. *Science*.

[23] Sun K., Geng X., Ji L. (2015). Exemplar component analysis: a fast band selection method for hyperspectral imagery. *IEEE Geoscience and Remote Sensing Letters*.

[24] Yu W., Wang Z., Li S. (2016). Hyperspectral image clustering based on density peaks and superpixel segmentation. *Journal of Image and Graphics*.

[25] Gong S., Zhang Y. (2016). Eddpc: an efficient distributed density center clustering algorithm. *Journal of Computer Research and Development*.

[26] Zhang Y., Chen S., Yu G. (2016). Efficient distributed density peaks for clustering large data sets in map reduce. *IEEE Transactions on Knowledge and Data Engineering*.

[27] Wu B., Wilamowski B. M. (2017). A fast density and grid based clustering method for data with arbitrary shapes and noise. *IEEE Transactions on Industrial Informatics*.

[28] Xu X., Ding S., Du M. (2016). Dpcg: an efficient density peaks clustering algorithm based on grid. *International Journal of Machine Learning and Cybernetics*.

[29] Xu X., Ding S., Sun T. A fast density peaks clustering algorithm based on pre-screening.

[30] Chen Y., Hu X., Fan W. (2019). Fast density peak clustering for large scale data based on KNN. *J/OL Knowledge-Based Systems*.

[31] Hou J., Pelillo M. A new density kernel in density peak based clustering.

[32] Liu Y., Ma Z., Yu F. (2017). Adaptive density peak clustering based on *K*-nearest neighbors with aggregating strategy. *Knowledge-Based Systems*.

[33] Chen J., He H. (2015). Research on density_based clustering algorithm for mixed data with determine cluster centers automatically. *Acta Automatic Sinica*.

[34] Wang X., Xu Y. (2017). Fast clustering using adaptive density peak detection. *Statistical Methods in Medical Research*.

